# Epidural Anesthesia versus General Anesthesia for Total Knee Arthroplasty: Influences on Perioperative Cognitive Function and Deep Vein Thrombosis

This article has been retracted.

**DOI:** 10.1155/2022/4259499

**Published:** 2022-09-10

**Authors:** Tao Ma, Guanhua Li, Hao Zhang, Yingxin Zhang, Lei Wang, Hailong Wu, Yang Chu, Xiaoli Zhao, Wei Wang

**Affiliations:** Department of Anesthesiology, PLA Rocket Force Characteristic Medical Center, Beijing 100088, China

## Abstract

**Purpose:**

This research mainly discussed the impacts of epidural anesthesia (EA) and general anesthesia (GA) on perioperative cognitive function (CF) and deep vein thrombosis (DVT) in patients undergoing total knee arthroplasty (TKA).

**Methods:**

One hundred and twenty-four patients undergoing TKA in our hospital between July 2015 and October 2021 were selected, of which 74 patients received EA (research group) and the other 50 patients received GA (control group). Perioperative CF, DVT, stress response indicators (norepinephrine, NE; cortisol, Cor), and heart rate (HR) levels were observed and compared. Risk factors affecting DVT of TKA patients were analyzed by logistic regression.

**Results:**

The research group had statistically better CF than the control group, with notably lower NE, Cor, and HR levels and incidence of DVT. Logistic regression analysis showed that the type of anesthesia and MoCA were risk factors for DVT in TKA patients.

**Conclusion:**

EA is more feasible for patients undergoing TKA, which is conducive to improving their CF, relieving stress responses, and reducing the incidence of DVT, with a certain sedative effect.

## 1. Introduction

With the aggravation of population aging, the elderly suffering from joint disease has become more and more common [1]. Osteoarthritis, as a commonly seen chronic disease in the elderly, has an increasing risk with age, which adversely affects the quality of life and retirement life of the elderly [2]. Total knee arthroplasty (TKA) is a surgical procedure that replaces the knee joint with artificial components and is commonly used to treat conditions such as osteoarthritis and rheumatoid arthritis [3]. According to epidemiological data, there were as many as 600,000 cases of TKA in the United States in 2012, and the number is expected to increase to 1.26 million cases per year by 2030, imposing a huge burden on the healthcare system [4]. TKA has been shown to be beneficial to relieve patients' pain and improve long-term function and life quality [5, 6]. However, this procedure is also accompanied by certain risk of complications, which may lead to postoperative cognitive dysfunction, deep vein thrombosis (DVT), and other adverse events [7, 8]. The causes of cognitive dysfunction or DVT after TKA are complicated, and the type of anesthesia is also an influencing factor that should not be underestimated [9]. This research mainly analyzes the impacts of epidural anesthesia (EA) and general anesthesia (GA) on cognitive function (CF) and DVT of TKA patients during the perioperative period, aiming at providing novel new insights for management optimization of such patients.

GA has favorable sedative and analgesic effects, but overdose of propofol and opioids may exert inhibitory effects on the central nervous system and respiratory system, which is not conducive to hemodynamic stability [10]. GA is also known to increase the risk of cerebrovascular adverse events [11]. And despite the inhibitory action of GA on the activity of cerebral cortex and hypothalamus, it may not be effective in inhibiting traumatic stress and inflammatory indicators, which may exert adverse effects on patients' CF and induce DVT [12]. EA, as a local anesthesia method, achieves anesthesia by injecting analgesics into the epidural space to block sensory nerves [13]. Such anesthesia not only induces vasodilation in the occluded area to increase blood flow but also preserves the patient's consciousness and provides pain relief [14, 15]. In the study of Zhu et al. [16], it was pointed out that EA significantly improved the CF of postoperative esophageal cancer patients than GA. Hafezi et al. [17] also reported that EA used in plastic surgery has a preventive effect on DVT.

Since there are few studies on the influences of GA and EA on CF and DVT in patients undergoing TKA during the perioperative period at present, this study mainly conducted in-depth analysis in this aspect and is hereby reported.

## 2. Data and Methods

### 2.1. General Data

This research has been approved by the Ethics Committee of PLA Rocket Force Characteristic Medical Center and was conducted in strict compliance with the Declaration of Helsinki. First, 124 patients undergoing TKA in the PLA Rocket Force Characteristic Medical Center from July 2015 to October 2021 were selected. Inclusion criteria are as follows: all patients were diagnosed by clinical and imaging examinations and met the surgical indications; patients and their families were clear about the purpose of this experiment and provided informed consent; American Society of Anesthesiologists (ASA) grade I-II [18]; and age > 18. Exclusion criteria are as follows: malignant tumors or severe heart, liver, and kidney diseases; mental disorders or mental illness; abnormal echocardiography (ECG) examination results; infectious diseases; previous treatment history for the disease; use of drugs in the last six months that might affect the experimental results; presence of DVT before surgery; and contraindications to anesthesia. The 124 patients with TKA were grouped according to anesthesia methods, with 74 receiving EA in the research group (RG) and 50 receiving GA in the control group (CG). The male to female ratio and mean age (years old) in RG were 41 : 33 and 59.50 ± 11.12, respectively, and the data in CG were 29 : 21 and 57.96 ± 8.18. RG and CG showed no evident differences in baseline data like gender and age (*P* > 0.05).

### 2.2. Anesthesia Methods

Both groups of subjects underwent TKA. After the preparation before anesthesia, CG received GA and RG received EA.

#### 2.2.1. GA

1.5-2.0 mg/kg propofol (Shanghai Yuanye Biotech, B33792-100 mg), 0.4 *μ*g/mL sufentanil (Sigma-Aldrich (Shanghai), S-008-1ML), 0.15-0.2 mg/kg cis-atracurium (Shenzhen Jianzhu Biotech, 30119630), and 30-50 *μ*g/kg midazolam (Nhwa Pharmaceutical Co. Ltd, China) were used for anesthesia induction. Then, endotracheal intubation and mechanical ventilation were performed. After successful anesthesia induction, continuous pumping of 15-75 *μ*g/kg·min propofol and 0.05-0.15 *μ*g/kg·min remifentanil (Sigma-Aldrich (Shanghai), R-024-1ML) was administered intraoperatively, accompanied by auxiliary inhalation of 1-2% sevoflurane (Shanghai Fuyu Biotech, FY23996-25) and intermittent addition of atracurium (Shanghai Yuanye Biotech, Y54583).

#### 2.2.2. EA

Epidural puncture of L3-4 was performed, and 5 mL 1.5% lidocaine (Shenzhen ChemStrong Scientific, L0595000) was added, followed by catheterization. 15 mL 0.5% ropivacaine (Beijing Biolab Biotech, BP0658-FKD) was given intraoperatively.

### 2.3. Endpoints

#### 2.3.1. CF

The evaluation was carried out through the Montreal Cognitive Assessment Scale (MoCA) [19]. The scale has a score ranged from 0 to 30 points, which was directly proportional to the patient's CF. The assessment was conducted before and 3 days after the surgery.

#### 2.3.2. Heart Rate (HR) Level

HR levels were measured at the following time points: before anesthesia (T1), 30 min after anesthesia (T2), end of surgery (T3), and 2 hours after surgery (T4).

#### 2.3.3. Stress Indexes

Norepinephrine (NE) and cortisol (Cor) of the subjects were detected at T1 and T4, using the corresponding human ELISA kits supplied by Shanghai Jianglai Industrial Limited By Share Ltd. The operation procedure strictly followed the instruction of human ELISA kits.

#### 2.3.4. DVT

The incidence of DVT was calculated by counting the cases of DVT after operation.

### 2.4. Statistical Processing

Statistical analysis was performed using SPSS22.0 (Beijing Easy Bio Technology), and the significance level was *P* < 0.05. A chi-square test was employed for intergroup comparisons of count data described in the form of number of cases/percentage (*n*/%), and the continuity correction chi-square test was adopted once the theoretical frequency of the chi-square test was <5. Mean ± SEM was used to represent measurement data; the differences between groups used the independent sample *t*-test, and those between two time points of the two groups adopted the paired *t*-test. Among them, the count data involved in this study included gender, surgical site, alcoholism, and smoking, and the measurement data included mean age, disease course, body mass index (BMI), and MoCA score. Logistic multivariate regression analysis was performed to identify risk factors of DVT in TKA patients.

## 3. Results

### 3.1. The Two Cohorts of Patients Undergoing TKA Showed Comparable Baseline Data

Of the 124 patients undergoing TKA, 50 cases receiving GA were included in CG and 74 cases receiving EA were included in RG. The two cohorts were similar in gender, average age, course of disease, BMI, operation site, operation time, duration of anesthesia, alcoholism, smoking, diabetes, hypertension, and other baseline data, with compatibility (*P* > 0.05) (Table 1).

### 3.2. The CF Is less Affected in Patients Receiving EA during TKA

CF was assessed using the MoCA scale, and no marked difference was found between RG and CG prior to anesthesia (*P* > 0.05); but the postanesthesia score was higher in RG than in CG, with statistical significance (*P* < 0.05) (Figure 1).

### 3.3. HR Level and Stress Response Changes Were Smaller in Patients Receiving EA during TKA

We evaluated the influence of two anesthesia methods on HR and stress response by measuring HR level and stress response. The data showed increased HR of the two groups at T2 and T3 compared with the value at T1; at T4, the HR level of RG was notably lower compared with T2 and T3, as well as the level of CG at T4, with statistical significance (*P* < 0.05). In terms of NE and Cor, their levels were similar in the two cohorts at T1 (*P* > 0.05), but increased markedly at T4 (*P* < 0.05), with significant differences between RG and CG at T4 (*P* < 0.05) (Figure 2).

### 3.4. The Incidence of DVT Was Lower in Patients Receiving EA during TKA

We recorded and compared the occurrence of DVT between groups to evaluate the influence of two anesthesia types on the incidence of DVT. DVT occurred in 12 cases in CG and 7 cases in RG, with an obvious lower incidence in RG compared with CG (9.46% vs. 24.00%, *P* < 0.05) (Figure 3).

### 3.5. Type of Anesthesia Is an Independent Risk Factor for DVT in TKA Patients

We included factors of differences (anesthesia type, MoCA, NE, Cor, and HR) into the analysis and assigned them as dependent variables for subsequent multivariate analysis with the logistic regression model, taking whether or not they affected the occurrence of DVT in TKA patients as the dependent variable. The results showed that the type of anesthesia (*P* < 0.001) and MoCA (*P* < 0.001) were independent risk factors for DVT in TKA patients (Table 2).

## 4. Discussion

For osteoarthritis, a common orthopedic disease with a sharp increase in the number of resulting fractures, TKA is undoubtedly an ideal treatment [20]. TKA is mostly performed in the elderly who are at an increased risk of perioperative cognitive dysfunction due to poor physical condition and fragile physiological function of the nervous system [21]. On the other hand, TKA patients may have varying degrees of coagulation function changes, which is one of the pathological causes of DVT [22]. This study mainly explores the influence of anesthesia on CF and DVT of TKA patients during the perioperative period.

Different anesthesia types have different effects on patients' nervous system and coagulation state, as well as CF and DVT [23]. Ishii et al. [24] also proposed that anesthesia may be a trigger for the need to prevent venous thromboembolism events. When the human body is under anesthesia, its cerebral blood flow will be reduced and the brain metabolism will be blocked, which may affect neuronal signaling [25]. GA can induce abnormal expression of brain memory protein level and serum central nervous system-specific protein S-100*β*, which would adversely affect patients' central nervous system, resulting in cognitive dysfunction [26], while EA has been shown to reduce the adverse effects on the central nervous system by lowering serum S-100*β* protein concentration, thus reducing the risk of postoperative cognitive dysfunction in elderly patients [10]. In our study, the MoCA score decreased statistically in both cohorts after anesthesia, with a markedly higher score in RG versus CG, suggesting that EA had little influence on the CF of TKA patients, which was consistent with the results of Ekblad [9]. Besides, we found deceased HR level at T4 in RG compared with T2 and T3 and CG at T4, as well as notably lower NE and Cor levels in RG versus CG at T4, indicating that EA had a sedative effect on TKA patients and could alleviate their stress responses. Consistently, Li et al. [27] reported a small impact of EA on patients' stress responses in thoracic surgery for esophageal cancer. Furthermore, we found a statistically lower incidence of DVT in RG compared with CG (9.46% vs. 24.00%), suggesting that EA can reduce the risk of DVT in TKA patients, which is similar to the findings of Hafezi et al. [17]. EA may reduce the risk of DVT development by preventing postoperative hypercoagulability, thus reducing postoperative thromboembolic complications [28]. Other studies have shown that under EA, anaesthetics are absorbed into the blood through the epidural space, which can inhibit the aggregation, release, and adhesion of platelets and improve the coagulation function of patients [29]. However, GA may activate platelet membrane glycoprotein and promote platelet aggregation, negatively influencing the body's coagulation function [29]. Finally, we conducted an in-depth exploration of the risk factors influencing the occurrence of DVT in TKA patients through logistic multivariate regression analysis. The results confirmed that the type of anesthesia and MoCA were independent risk factors for DVT in TKA patients. It has also been suggested that in order to prevent DVT after TKA, preoperative risk assessment of comorbidities in patients can be considered [30].

The novelty of this study is as follows: first, combined with indicators such as CF, HR, stress response, and incidence of DVT, it is confirmed that EA has a small impact on patients' CF during TKA and can help prevent DVT to a certain extent. Second, the logistic regression model was used for multivariate analysis, which proved that anesthesia type and MoCA were independent risk factors for DVT in TKA patients, further emphasizing the importance of anesthesia management for DVT prevention in TKA patients. But still, this research has some limitations. First of all, this is a retrospective instead of a blind or randomized study, which may lead to reporting bias. Second, this is a single-center small sample study, so the universality and accuracy of the research results may be affected to some extent. Third, inflammation, oxidative stress, and coagulation indexes were not included in the analysis, nor was there supplementary follow-up to analyze the long-term CF, DVT, and other complications of patients under the two anesthesia methods. The above deficiencies will be gradually addressed in the future.

## 5. Conclusion

To sum up, compared with GA, EA has less influence on perioperative CF and DVT of TKA patients, with high clinical application and popularization value.

## Figures and Tables

**Figure 1:** Cognitive function of TKA patients. ^∗∗^*P* < 0.01. Paired *t*-test was used to analyze the measurement data between groups before and after the intervention.

**Figure 2:** Stress response and HR level of TKA patients. (a) The HR level of TKA patients in both groups increased significantly at T2 and T3, and the HR level in the research group was lower than that in the control group at T4. (b) The NE level of TKA patients in both groups increased significantly at T4, with a lower level in the research group. (c) The Cor level of TKA patients in both groups increased significantly at T4, with a lower level in the research group. Note: ^∗∗^*P* < 0.01. Paired *t*-test was used to analyze the measurement data between groups before and after the intervention.

**Figure 3:** DVT in TKA patients. Chi-square test was used to analyze the incidence of DVT in both groups.

**Table 1:** Baseline data of patients undergoing TKA (*n*, mean ± SEM).

Factor	Control group (*n* = 50)	Research group (*n* = 74)	*χ* ^2^/*t*	*P*
Gender (male/female)	29/21	41/33	0.082	0.775
Average age (years old)	57.96 ± 8.18	59.50 ± 11.12	0.838	0.404
Course of disease (years)	9.26 ± 2.27	10.04 ± 2.99	1.564	0.120
BMI (kg/m^2^)	25.89 ± 4.03	26.01 ± 5.16	0.035	0.973
Surgical site (unilateral/bilateral)	26/24	32/42	0.919	0.338
Operation time (min)	99.78 ± 28.38	95.92 ± 31.69	0.694	0.489
Duration of anesthesia (min)	145.62 ± 39.18	141.49 ± 44.63	0.531	0.597
Alcoholism (yes/no)	30/20	36/38	1.544	0.214
Smoking (yes/no)	28/22	35/39	0.904	0.342
Diabetes (with/without)	23/27	32/42	0.092	0.762
Hypertension (with/without)	25/25	34/40	0.197	0.658

**Table 2:** Multivariate analysis of factors affecting the occurrence of DVT in TKA patients.

Characteristic	Class	OR	95% CI	*P*
Anesthesia type	EA vs. GA	0.012	0.002-0.085	<0.001
MoCA	Continuous variable	0.516	0.373-0.713	<0.001
NE	Continuous variable	1.216	0.048-30.538	0.906
Cor	Continuous variable	1.691	0.062-46.102	0.755
HR	Continuous variable	1.014	0.965-1.066	0.585

## Data Availability

The labeled datasets used to support the findings of this study are available from the corresponding author upon request.
